# Therapeutic Endoscopic Interventions in Choledocholithiasis: Efficacy of Endoscopic Retrograde Cholangiopancreatography

**DOI:** 10.7759/cureus.76955

**Published:** 2025-01-05

**Authors:** Mohmad Sejarali Sayeed, Shivam Sharma, Jay Prakash S Rajput, Dhvani Shah, Sajidali S Saiyad, Tehsin Saiyad, Nehal Shah, Chetan Kumar R

**Affiliations:** 1 Surgical Gastroenterology, Aryavart Hospital, Meerut, IND; 2 Surgery, Jaya Maxwell Hospital, Haridwar, IND; 3 Physiology, Pacific Medical College and Hospital, Udaipur, IND; 4 Pediatric Surgery, B.J. Medical College and Civil Hospital, Ahmedabad, IND; 5 Microbiology, Veer Narmad South Gujarat University, Surat, IND; 6 Pharmacology, Dr. M.K. Shah Medical College and Research Centre, Ahmedabad, IND; 7 Forensic Medicine, Rajmata Vijaya Raje Scindia Medical College, Bhilwara, IND

**Keywords:** biliary stone removal, choledocholithiasis management, endoscopic retrograde cholangiopancreatography (ercp), endoscopic sphincterotomy (es), therapeutic endoscopy

## Abstract

Introduction: Choledocholithiasis, a condition characterized by stones in the common bile duct (CBD), frequently results in obstructive jaundice and associated complications. Endoscopic retrograde cholangiopancreatography (ERCP) has emerged as the gold standard for treating this condition, offering a minimally invasive therapeutic approach. However, while ERCP is widely used, its efficacy in managing diverse clinical presentations and potential complications necessitates further investigation. Additionally, data on ERCP's effectiveness in various clinical scenarios, particularly concerning stone size and location, remain inconsistent, highlighting the need for more comprehensive research in this area.

Objective: This study aims to evaluate the effectiveness of ERCP as a therapeutic intervention for choledocholithiasis, focusing on procedural outcomes, stone clearance rates, and associated complications.

Methods: A retrospective study was conducted on 50 patients diagnosed with choledocholithiasis who underwent ERCP at a tertiary care hospital between January 2022 and December 2023. Data on patient demographics, clinical presentation, imaging, laboratory findings, and procedural outcomes were collected. ERCP procedures, including endoscopic sphincterotomy (ES) with balloon extraction and stenting, were performed by experienced endoscopists. Statistical analysis was done using SPSS version 25.

Results: The majority of patients were aged 31-70 years, with abdominal pain (96%) being the most common symptom. ERCP successfully cleared the CBD in 76% of cases in a single session, with repeat ERCP required for 18% of patients. Complications occurred in 20% of cases, with pancreatitis (10%) being the most common. Smaller stones (≤10 mm) had higher success rates for single-session clearance, while larger stones (>15 mm) often required repeat procedures or surgery. Distal CBD stones were cleared more effectively compared to those in proximal locations.

Conclusion: ERCP remains an effective and safe treatment for choledocholithiasis, particularly for smaller and distal CBD stones. The procedure's safety and efficacy support its continued use as the gold standard for managing choledocholithiasis.

## Introduction

Endoscopic retrograde cholangiopancreatography (ERCP) plays a pivotal role in the therapeutic management of choledocholithiasis, a condition characterized by the presence of stones in the common bile duct (CBD), which frequently leads to complications such as obstructive jaundice, abdominal pain, and skin yellowing [1,2]. Initially developed as a diagnostic tool, ERCP has undergone significant advancements, evolving into a combined diagnostic and therapeutic procedure that minimizes the need for invasive surgeries like open choledochotomy, as highlighted by Maple JT et al. (2011) and Dasari et al. (2013) [3,4]. Its integration with endoscopic sphincterotomy (ES) facilitates effective stone extraction and bile duct decompression, enhancing recovery and reducing morbidity [4].

Despite its widespread adoption and effectiveness, ERCP's precise advantages and limitations compared to alternative surgical approaches, particularly laparoscopic procedures, remain areas of ongoing investigation. Recent studies, such as Zhang et al. (2023), have demonstrated the superiority of ERCP over laparoscopic surgery in specific contexts, especially among post-cholecystectomy patients, highlighting its role in improving patient outcomes and recovery times [5,6]. Similarly, Ödemiş et al. (2016) underscored the challenges associated with managing complex or large bile duct stones and emphasized the niche ERCP occupies in addressing these scenarios without resorting to more invasive interventions [2]. The procedure is particularly recommended for patients with high-risk profiles, such as those presenting with elevated bilirubin levels or significant bile duct dilation [7].

However, ERCP is not without complications, including risks of post-procedure pancreatitis, bleeding, and cholangitis [8]. Advances in technique, such as the use of stents and incorporation of non-invasive imaging modalities like magnetic resonance cholangiopancreatography (MRCP), have been pivotal in mitigating these risks and enhancing the safety profile of ERCP [5].

This study aims to address the gap in understanding the role of ERCP in specific high-risk populations and complex clinical scenarios, positioning ERCP as a cornerstone of modern biliary management. Focusing on patient outcomes and procedural efficacy, this research seeks to solidify the link between ERCP's objectives of minimally invasive, effective, and safe management of choledocholithiasis and its demonstrated clinical advantages, as highlighted in the conclusions [9,10].

## Materials and methods

This retrospective cohort study analyzed patients with choledocholithiasis who underwent ERCP at a tertiary care hospital in Surat between January 2022 and December 2023. Data were obtained from medical records, including patient demographics, clinical presentation, imaging findings, laboratory results, and procedural outcomes. The study was approved by the institutional review board (IRB) (Approval No. 26062021), and all patient data were anonymized to maintain confidentiality.

The study included 50 patients based on the sample size calculation described earlier, which was determined using an estimated effect size derived from prior studies on ERCP outcomes in choledocholithiasis, as reported in the works of Dasari et al. (2013), Zhang et al. (2023), and Pereira-Lima et al. (1998) [4,5,10]. The primary outcome of interest was the successful clearance of stones from the CBD, influenced by factors such as stone size. Based on previous literature, the expected success rates for CBD clearance were assumed to be 90% for patients with small stones (≤10 mm) and 60% for patients with larger stones (>10 mm). To quantify the magnitude of the difference in success rates between these two groups, Cohen's h was calculated, resulting in a value of 0.73, indicating a moderate to large effect size. This suggests that the difference in success rates between small and large stones is substantial and could be detected with high statistical power.

The sample size was calculated using a significance level (alpha) of 0.05 and a power of 80%, standard parameters for ensuring the detection of meaningful effects in clinical studies. The calculated sample size of 50 patients was sufficient to detect a clinically significant difference between the groups with adequate statistical power, thus providing valid conclusions about the primary outcome.

This sample size also allowed for detecting differences in secondary outcomes, such as the need for repeat ERCP sessions and the incidence of complications (e.g., pancreatitis, cholangitis, bleeding), ensuring that the study was adequately powered to analyze both categorical and continuous variables.

The study included 50 adult patients (≥18 years) diagnosed with choledocholithiasis and undergoing therapeutic ERCP. Patients who met the inclusion criteria from the tertiary hospital's medical records database were considered for the study. Exclusion criteria were as follows: Patients with contraindications for ERCP (e.g., uncorrectable coagulopathies, severe cardiopulmonary instability, or active infection), as well as those with incomplete data or insufficient follow-up (less than 30 days post-procedure). ERCP was performed under sedation by an experienced endoscopist. Procedures included CBD cannulation, stone retrieval via baskets or balloon catheters, and biliary stenting if necessary. Outcomes were assessed based on stone clearance, procedural time, and complications within 30 days.

Data were analyzed using SPSS version 25. Continuous variables were expressed as mean ± SD, and categorical data as percentages. The chi-square test was used to compare categorical variables, and the Student's t-test was applied for continuous variables. A p-value of less than 0.05 was considered statistically significant. Subgroup analyses were performed based on stone size, CBD diameter, and the location of the calculus (distal/proximal CBD).

## Results

The study included 50 patients diagnosed with choledocholithiasis who underwent therapeutic ERCP. The patients' ages ranged from 27 to 81 years, with a mean age of 48.2 years (SD=13.18 years), with the majority (90%) falling between 31 and 70 years. Out of the 50 patients studied, 12 fell into the 31-40 age group, representing 24% of the total cases. This age group had the highest incidence of choledocholithiasis among all age groups in the study. Females slightly outnumbered males, with 54% of the patient population being female.

Abdominal pain was the most common symptom (96%), followed by jaundice (80%), vomiting (78%), and fever (74%). Itching and clay-colored stools were less frequent (14% and 12%, respectively). Laboratory findings showed elevated serum bilirubin in 42% of patients (above 6 mg%) and high alkaline phosphatase in 90%, indicating biliary obstruction due to stones.

All patients exhibited CBD dilatation, confirmed via ultrasonography and ERCP. Most patients (44%) had a CBD diameter between 10-12 mm, and 50% had stones sized 6-10 mm. Distal CBD stones were the most common (50%).

Endoscopic sphincterotomy (ES) with balloon extraction was the most common therapeutic intervention, performed in 36 out of 50 cases (72%). Stenting without stone extraction was conducted in 11 patients (22%), while basket retrieval was used in two cases (4%). Overall, 38 patients (76%) achieved common bile duct (CBD) clearance in a single session. Nine patients (18%) were required to repeat ERCP for complete clearance, while three patients (6%) with stones larger than 15 mm were referred for surgery.

The detailed outcomes and complications associated with the ERCP procedures are summarized in Table 1. It outlines the procedures performed, the percentage of successful CBD clearance, the need for repeat ERCP, and the complications observed, including pancreatitis, cholangitis, bleeding, and sepsis. The total complication rate was 20%, with post-ERCP pancreatitis being the most frequent, affecting 10% of patients. Cholangitis and bleeding occurred in 4% each. Sepsis, although rare, developed in one patient (2%), which proved fatal. Importantly, there were no cases of bile duct injury or retroduodenal perforation, which highlights the procedure's safety.

**Table 1:** ERCP procedure, outcomes, and complications ERCP: Endoscopic retrograde cholangiopancreatography; ES: Endoscopic sphincterotomy

	Parameters	Number of Patients	Percentage (%)
Procedure	ES with balloon extraction	36	72%
	ES with Basket retrieval	2	4%
	ES with stenting only	11	22%
	Sphincterotomy alone	0	0%
	Others	1	2%
Outcome	Successful CBD clearance	38	76%
	Repeat ERCP	9	18%
	Referred for surgery	3	6%
Complications	Pancreatitis	5	10%
	Cholangitis	2	4%
	Bleeding	2	4%
	Sepsis	1	2%
	Bile duct injury	0	0%
	Retroduodenal perforation	0	0%

The outcomes based on various parameters such as CBD diameter, stone size, and the site of calculus, emphasizing the significant impact of stone size on the procedure's success, are described in Table 2. Percentages are given with "n" denoting the number of patients for each group. CBD diameter and stone size are measured in millimeters. Stone size (≤10 mm) and the location of the calculus (distal) were significantly associated with successful CBD clearance (χ2=39.64, p<0.05), while CBD diameter did not have a significant effect (χ2=12.127, p>0.05). Stones measuring 6-10 mm were the most common, found in 25 patients (50%), followed by stones ≤5 mm in 14 patients (28%), stones >10-15 mm in nine patients (18%), and stones >15 mm in two patients (4%). Among the nine patients with stones sized >10-15 mm, none achieved successful clearance in a single ERCP session. Most of these patients (88.89%, 8/9) required a repeat ERCP for complete clearance, while 11.11% (1/9) ultimately required surgical intervention. Additionally, stones located in the distal CBD were cleared more successfully than those in proximal or multiple locations within the CBD.

**Table 2:** Outcome based on the parameter, stone size, and location post-ERCP CBD: Common bile duct; ERCP: Endoscopic retrograde cholangiopancreatography

Parameter	Outcome	Successful Clearance	Repeat ERCP	Surgery
CBD Diameter (8-10 mm)	Not Significant (p > 0.05)	86.67% (13/15)	13.33% (2/15)	0%
CBD Diameter (>10-12 mm)	Not Significant (p > 0.05)	68.18% (15/22)	31.82% (7/22)	0%
Stone Size (≤10 mm)	Significant (p < 0.05)	100% (14/14)	0%	0%
Stone Size (>15 mm)	Significant (p < 0.05)	0%	0%	100% (2/2)
Site of Calculus (Distal)	Not Significant (p > 0.05)	92% (23/25)	8% (2/25)	0%

## Discussion

This study highlights the significant role of ERCP in managing choledocholithiasis, particularly its effectiveness based on CBD conditions and stone characteristics. The results indicated a predominance of females (27 patients, 54%), with the highest incidence occurring in the 31-40 age group (12 patients, 24%). These findings are consistent with the general prevalence of choledocholithiasis observed in many populations, though this study did not directly compare with other demographic groups. The most common presenting symptoms were abdominal pain (48 patients, 96%), jaundice (40 patients, 80%), and vomiting (39 patients, 78%), aligning with the typical presentation of obstructive jaundice caused by CBD stones. These results corroborate previous studies on the common clinical presentation of choledocholithiasis, as reported by Ödemiş et al. (2016) and Maple JT et al. (2011) [2,3]. Laboratory results confirmed these clinical findings, with 21 patients (42%) exhibiting elevated bilirubin levels (>6 mg%) and 45 patients (90%) showing increased alkaline phosphatase levels, typical of biliary obstruction due to CBD stones. These findings are consistent with studies by Maple JT et al. (2011) and Pereira-Lima et al. (1998), further validating the diagnostic criteria used in this study [3,10].

ERCP was predominantly used for endoscopic sphincterotomy (ES) with balloon extraction, which was effective in 38 patients (76%) for CBD clearance in a single session. These findings are supported by previous studies that reported high success rates for endoscopic management of choledocholithiasis, with Ashton and McNabb (1998) achieving a 98% clearance rate, consistent with the results of Manes et al. (2019) and Dasari et al. (2013) [4,11,12]. However, larger stones (>15 mm) frequently required repeat ERCP sessions or surgical referral in 3 patients (6%), echoing the findings of ElGeidie (2014), who noted that large stones often necessitate additional interventions for complete clearance [1].

The complication rate in our study was 10 patients (20%), with pancreatitis being the most common complication affecting 5 patients (10%), followed by cholangitis and bleeding, each occurring in 2 patients (4%). These rates are similar to those reported in previous studies on ERCP, indicating the typical risks associated with the procedure. Notably, no bile duct injuries or perforations were observed in our cohort, which is consistent with the safety profile of ERCP when performed by experienced clinicians, as highlighted in other studies.

Our findings regarding stone size and location align with previous research, showing that smaller stones (≤10 mm) and those located in the distal CBD are more likely to be cleared successfully with a single ERCP session. All 14 patients with stones ≤10 mm achieved 100% clearance in a single session, while 23 patients (92%) with distal CBD stones were successfully cleared. This granular breakdown offers clinicians more precise guidance on expected outcomes based on stone characteristics. Despite the overall high success rate, larger stones or those located in more difficult locations (e.g., proximal CBD) require careful preoperative assessment and often additional interventions or surgery. This reinforces the importance of personalized treatment strategies for patients with complex choledocholithiasis, as emphasized in several studies, including Zhang et al. (2023) [5]. Our study also underscores ERCP's role as a first-line treatment for choledocholithiasis, particularly in high-risk surgical patients. The successful CBD clearance in 38 patients (76%) in a single session supports its use over surgical methods in many cases, as demonstrated in randomized trials.

Interestingly, our study found that CBD diameter did not significantly affect clearance success rates, contrasting with some previous assumptions. This finding warrants further investigation and may have implications for pre-procedure planning and patient selection.

The highest incidence of choledocholithiasis in the 31-40 age group (12 patients, 24% of cases) is a notable finding that may inform targeted screening and prevention strategies. This age-specific data contributes to the growing body of evidence on risk factors and demographic patterns in choledocholithiasis. 

This study on choledocholithiasis treatment using ERCP has several limitations that warrant consideration. The retrospective design introduces potential biases and data gaps, affecting result interpretation and generalizability. The reliance on existing medical records may have led to incomplete or inconsistent data collection. The sample size of 50 patients, while sufficient for primary outcome analysis, may limit external validity, particularly for rare complications or atypical presentations. The absence of long-term follow-up data prevents a comprehensive assessment of biliary symptom recurrence and sustained procedural efficacy. The study's focus on immediate and short-term outcomes (up to 30 days post-procedure) may not reflect the full spectrum of ERCP's long-term benefits and potential complications. The single-center nature of the study may limit generalizability to other healthcare settings with different patient populations, expertise levels, or equipment availability. These limitations underscore the need for prospective studies with larger cohorts and extended follow-up periods to validate the findings and provide more definitive evidence on long-term ERCP outcomes in choledocholithiasis treatment. Future research should address these constraints to enhance the robustness and clinical applicability of the results in guiding choledocholithiasis management strategies. Interestingly, the study found that CBD diameter did not significantly affect clearance success rates, contrasting with some previous assumptions and warranting further investigation. 

## Conclusions

This study highlights the efficacy and safety of ERCP as a therapeutic intervention for choledocholithiasis, particularly in managing small and distally located stones. The findings reinforce ERCP's role as a highly effective first-line treatment, often preferred over surgical interventions, especially in high-risk surgical patients. ERCP demonstrated substantial success in achieving bile duct clearance, particularly through endoscopic sphincterotomy with balloon extraction, while providing valuable insights into how stone size and location influence procedural outcomes. These results emphasize the procedure's effectiveness in minimizing invasive surgical interventions and enhancing patient outcomes.

The study also provides a critical analysis of complications associated with ERCP. While the overall safety profile was consistent with previous literature, complications such as pancreatitis, cholangitis, and bleeding were observed, underscoring the importance of skilled procedural execution and post-procedure monitoring. The absence of major injuries, such as bile duct perforation, highlights the safety of ERCP when performed by experienced clinicians. Despite these strengths, the study's retrospective design and lack of long-term follow-up underscore the need for larger, prospective studies to validate these findings, further explore risk factors for complications, and enhance long-term management strategies for choledocholithiasis.
